This article has been retracted.

# The causal effect of atopic dermatitis on lung cancer: A Mendelian randomization study

**DOI:** 10.1111/srt.13841

**Published:** 2024-07-04

**Authors:** Peng Huang, Feng Wen, QiuJi Wu, PengFei Zhang, Qiu Li

**Affiliations:** ^1^ Division of Abdominal Tumor Multimodality Treatment Cancer Center West China Hospital Sichuan University Chengdu Sichuan China; ^2^ Department of Medical Oncology Cancer Center West China Hospital Sichuan University Chengdu Sichuan China; ^3^ Department of Radiation Oncology Cancer Center West China Hospital Sichuan University Chengdu Sichuan China; ^4^ Gastric Cancer Center Division of Medical Oncology Cancer Center West China Hospital Sichuan University Chengdu Sichuan China

**Keywords:** atopic dermatitis, lung cancer, Mendelian randomization, single nucleotide polymorphisms

## Abstract

**Background:**

Growing evidence has shown that atopic dermatitis (AD) may decrease lung cancer (LC) risk. However, the causality between the two diseases is inconsistent and controversial. Therefore, we explored the causal relationship between AD and different histological subtypes of LC by using the Mendelian randomization (MR) method.

**Materials and methods:**

We conducted the MR study based on summary statistics from the genome‐wide association studies (GWAS) of AD (10,788 cases and 30,047 controls) and LC (29,266 cases and 56,450 controls). Instrumental variables (IVs) were obtained after removing SNPs associated with potential confounders. We employed inverse‐variance weighted (IVW), MR‐Egger, and weighted median methods to pool estimates, and performed a comprehensive sensitivity analysis.

**Results:**

The results of the IVW method suggested that AD may decrease the risk of developing lung adenocarcinoma (LUAD) (OR = 0.91, 95% CI: 0.85‐0.97, *P* = 0.007). Moreover, no causality was identified between AD and overall LC (OR = 0.96, 95% CI: 0.91–1.01, *P* = 0.101), lung squamous cell carcinoma (LUSC) (OR = 1.04, 95% CI: 0.96–1.036, *P* = 0.324), and small cell lung carcinoma (SCLC) (OR = 0.95, 95% CI: 0.82–1.10, *P* = 0.512). A comprehensive sensitivity test showed the robustness of our results.

**Conclusion:**

The present study indicates that AD may decrease the risk of LUAD in the European population, which needs additional investigations to identify the potential molecular mechanisms.

## 1 INTRODUCTION

Lung cancer (LC) is among the most prevalent types of cancer and ranks the leading cause of cancer‐related death globally, with an annual of roughly 2,206,771 new cases and 1,796,144 deaths.^1^ In the past decade, the development of molecularly targeted therapy and immunotherapy significantly improves survival outcomes.^2^ According to statistics, the 3‐year relative survival rate of LC patients increased from 22% to 33%.^3^ Additionally, low‐dose computed tomography (LDCT) is recommended for LC screening in asymptomatic individuals. However, LDCT is plagued by several challenges such as false‐positive errors, radiation hazards, and insufficient resources for performing routine screening.^4^ In the US, only 5% of high‐risk individuals have used LDCT for screening, which has significantly impeded the early diagnosis of LC.^4^, ^5^, ^6^ Regarding the heavy disease burden of LC, an initiative to improve the understanding of potential risk factors and disease pathological development for establishing surveillance programs and screening high‐risk populations of LC is ongoing,^7^ which might significantly improve the prognosis of patients.

Atopic dermatitis (AD), also known as eczema, is the most prevalent form of inflammatory dermatosis, characterized by itchy and relapsing eczematous skin.^8^ The incidence of AD has steadily increased in the past few decades, affecting up to 15%−20% of people in Europe.^9^ The disease burden of AD ranks fifteenth among nonfatal conditions with respect to disability‐adjusted life‐years.^10^ AD is associated with psychiatric morbidities, sleep disruption, as well as decreased quality of life, which impose remarkable psychosocial burdens on patients and their families.^11^ Although the pathogenesis of AD is not fully understood, existing evidence has shown that genetic susceptibility,^12^ impaired epithelial barrier,^13^ deregulated immune system and skin microbiota dysbiosis^14^ are key factors in the onset of AD.

Given the remarkable disease burden of LC and the growing AD prevalence,^7^, ^8^ the comorbidities of both conditions may be more common. Previous epidemiological studies have suggested that AD was associated with cancer incidence, and most indicated that it may increase the risk of certain types of cancers compared with the non‐AD population.^15^, ^16^ In recent decades, there have been several studies regarding the association between AD and LC risk, however, findings on the causality between both diseases remain controversial. Previous meta‐analyses and several observational studies have shown that AD was associated with a decreased risk of LC compared to the non‐AD population.^15^, ^17^, ^18^, ^19^ Nonetheless, several large‐scale population‐based studies found no statistically significant evidence of lower LC risk in the AD population.^20^, ^21^, ^22^ Besides, unmeasurable confounding factors of observational studies are unavoidable and may result in biases, which affect the reliability of results. Randomized controlled trial (RCT) is regarded as the standard methodology for investigating the causal association of certain risk factors on disease development.^23^, ^24^ Nonetheless, RCTs are not always practical owing to high expense or ethical problems.^23^

Mendelian randomization (MR) is an emerging method to examine causal relationships between risk factors and disease outcomes.^25^ It employs single nucleotide polymorphisms (SNPs) robustly correlated with risk factors as genetic instrumental variables (IVs) to mimic the RCT setting, thereby avoiding reverse causality and various biases from confounding in observational studies.^25^, ^26^ In this study, we conducted the MR study to explore the causal effect of genetically predicted AD on the risk of LC, aiming to provide novel insights into the mechanism of AD affecting the pathological development of LC and a theoretical basis for the clinical management of LC.

## 2 MATERIALS AND METHODS

### 2.1 Study design and data resources

A two‐sample MR study was implemented by a basic scheme of MR analysis. Three principal assumptions of the MR study were met: IVs were robustly associated with exposure; IVs were not affected by confounding factors; IVs only affected the outcome through exposure^25^ (Figure 1).

**FIGURE 1:** The schematic illustration of the MR study to explore the causal relationship between atopic dermatitis and lung cancer.

For genetically predicted AD, we retrieved the Genome‐wide association study (GWAS) summary data from the EArly Genetics and Life Course Epidemiology (EAGLE) consortium^27^ via the Integrative Epidemiology Unit‐OpenGWAS project online platform (accessible at https://gwas.mrcieu.ac.uk/ GWAS ID: ieu‐a‐996). The GWAS of the EAGLE consortium covered 20 independent studies comprising a total of 10,788 cases and 30,047 controls.^27^ For LC, we retrieved the GWAS summary data from a large‐scale aggregated study that included a total of 29,266 cases and 56,450 controls with European ancestry.^28^ This study conducted a meta‐analysis with an inverse‐variance weighted (IVW) approach based on summary data of several previously reported LC GWAS studies of European populations: the OncoArray series, IARC, SLRI, NCI, ICR, MDACC, Harvard, Germany and deCODE.^28^ It also subcategorized LC cases by histological strata: lung adenocarcinoma (LUAD), lung squamous cell carcinoma (LUSC), and small cell lung carcinoma (SCLC).^28^ Detailed information on GWAS studies of AD and LC is shown in Table 1.

**TABLE 1:** Detail information of the data for the cohort population.

Disease	Number of cases	Number of controls	Population	Resource/Reference
AD	10788	30047	European	25
LC	29266	56450	European	26
LUSC	7426	55627	European	26
LUAD	11273	55483	European	26
SCLC	2664	21444	European	26

### 2.2 Selection of genetic IVs

Since few SNPs identified by AD GWAS have achieved a genome‐wide significance threshold (*P* < 5E‐08). We used a relaxed threshold (*P* < 5E‐06) to select SNPs. Furthermore, to eliminate linkage disequilibrium (LD) caused by AD‐related SNPs, we performed structural clumping at a strict threshold of LD, *R* ^2^ < 0.001, and genetic distance <10000 kb based on estimates from European samples in the 1,000 Genomes Project.^29^ To guarantee the IVs were independent of confounding factors, we used the PhenoScanner V2 database (http://www.phenoscanner.medschl.cam.ac.uk/) at the threshold (*P* = 5E‐08, proxy: EUR, *R* ^2^ = 0.8, Build = 37) to remove SNPs correlated with cofounders.^30^ Then, we used the F‐statistic (F = Beta2/Se2) to avoid weak instrument bias and SNPs with F‐ statistic less than 10 were removed, which might ensure the significant association between IVs and AD.^31^, ^32^ After the strict screening, SNPs associated with AD were used as IVs and we extracted them from datasets of LC and its histological subtypes for subsequent MR analysis.

### 2.3 MR analysis

In our study, three MR analytical methods including IVW, MR‐Egger, and weighted median (WM) were employed to assess the causality of AD and LC.^33^ The preliminary MR analysis was performed by adopting the IVW method, which could gain an aggregated causal estimate between exposure and outcome and provide the highest statistical power.^34^ Therefore, IVW was conducted as the primary approach to infer preliminary associations of AD with LC. Moreover, another two methods, MR‐Egger and WM, were deployed as complements to test the causal association. A two‐sided *P* < 0.05 was considered suggestive association and a *P* < 0.017 (Bonferroni correction *P* = 0.05/3 outcomes) was deemed as statistically significant.

### 2.4 Sensitivity analysis

In order to ensure the robustness of the preliminary analysis, several approaches were employed to detect the presence of heterogeneity and horizontal pleiotropy. In this study, heterogeneity was assessed by Cochran's Q test.^35^ It was considered as an absence of heterogeneity in the causal inference when Q‐statistic‐derived *P* > 0.05. The funnel plot was also utilized to test the heterogeneity.^29^ Additionally, we performed the pleiotropy test by using the MR‐Egger method and MR pleiotropy residual sum and outlier (MR‐PRESSO) test.^36^, ^37^ It was regarded as having no directional pleiotropic effect between AD and LC when there was an absence of a statistically significant intercept term of the MR‐Egger regression.^37^ Horizontal pleiotropy was evaluated by MR‐PRESSO test and it could be adjusted with outlier removal.^38^ Finally, we conducted the leave‐one‐out test to assess whether our MR analysis was affected by particular SNPs.^39^

All MR analyses were performed by R software (version 4.1.2) and several R packages including the “TwoSampleMR,” “MR‐PRESSO,” and “forestplot” were used for statistical analyses and results visualization.

## 3 RESULTS

### 3.1 Strength of genetic instruments

Based on the above selecting threshold for IVs, a total of 39 SNPs significantly associated with AD were obtained, and after further screening by the PhenoScanner v2 database, 14 SNPs associated with potential confounding factors were removed, as shown in Table 2. Finally, 25 SNPs were used as IVs for subsequent analysis (Table 3). The F‐statistics of included SNPs were above 10, suggesting that selected IVs were significantly associated with AD and would not be affected by weak instrument bias. Then, we extracted SNPs from datasets of LC and its pathological subtypes, and finally, SNPs related to overall LC, LUSC, LUAD, and SCLC were extracted for subsequent analysis.

**TABLE 2:** The detailed contents of SNPs associated with potential confounding factors.

SNP	Trait	EA	OA	*P*	Source (PMID)
rs2212434	Asthma	C	T	1.22E‐47	UKBB
rs13266315	Asthma	A	G	1.43E‐08	29273806
rs13419662	Asthma	A	G	1.29E‐11	UKBB
rs12144049	Asthma	C	T	2.65E‐11	UKBB
rs2041733	Asthma	C	T	9.73E‐11	UKBB
rs479844	Asthma	G	A	3.05E‐10	UKBB
rs7700687	Asthma	C	T	6.43E‐09	UKBB
rs6062486	Inflammatory bowel disease	A	G	6.08E‐14	26192919
rs6419573	Inflammatory bowel disease	C	T	2.18E‐09	26192919
rs2581790	Self‐reported gout	C	T	1.60E‐10	UKBB
rs188557945	Self‐reported interstitial lung disease	A	G	2.18E‐09	UKBB
rs4976685	Chronic kidney disease	A	G	1.30E‐08	26831199
rs10790275	Rheumatoid arthritis	C	G	7.00E‐14	24390342
rs4151657	Vascular or heart problems diagnosed by doctor: high blood pressure	C	T	5.37E‐12	UKBB

**TABLE 3:** Detail information on instrumental variables of atopic dermatitis.

SNP	EA	OA	EAF	BETA	SE	*P*‐value	F
rs906363	C	T	0.147634	0.112244	0.0233251	1.52E‐06	23.15683715
rs11581328	A	G	0.20783	−0.116874	0.0229406	3.56E‐07	25.95531303
rs8006	C	G	0.387951	0.0854077	0.0171394	6.37E‐07	24.83149254
rs3120745	G	A	0.690562	−0.106987	0.0195755	4.73E‐08	29.87007356
rs181628386	C	T	0.012653	0.47516	0.100704	2.42E‐06	22.26313423
rs280729	G	A	0.182003	0.105335	0.0218012	1.38E‐06	23.34450132
rs144143913	G	A	0.015207	0.452815	0.0931278	1.18E‐06	23.64192976
rs13152362	A	G	0.206489	−0.116523	0.0214189	5.45E‐08	29.59572535
rs12188917	C	T	0.205033	0.170064	0.0215238	2.89E‐15	62.42907262
rs11738721	A	G	0.422463	−0.095364	0.0179028	1.02E‐07	28.37442034
rs12334935	A	G	0.473769	0.0926111	0.0168776	4.18E‐08	30.10958055
rs145009390	G	C	0.021662	0.328182	0.0679122	1.37E‐06	23.35252876
rs79030114	T	A	0.024846	0.307702	0.0661004	3.29E‐06	21.66967825
rs13302629	A	G	0.250947	−0.0985361	0.0215207	4.75E‐06	20.96418345
rs61850526	T	C	0.029934	0.273618	0.0550251	6.73E‐07	24.72678469
rs11256611	A	C	0.125131	0.114025	0.0248019	4.34E‐06	21.13636293
rs2433192	A	G	0.519422	−0.0873875	0.0169757	2.69E‐07	26.49983971
rs1496701	T	C	0.014795	0.749778	0.162318	3.91E‐06	21.33693433
rs4913279	C	T	0.631334	0.081698	0.0174638	2.94E‐06	21.88493957
rs1038165	T	C	0.562112	0.079396	0.0169963	3.04E‐06	21.82169442
rs11156881	T	C	0.23906	−0.10883	0.0219665	7.39E‐07	24.54570604
rs111375762	G	T	0.043373	0.263773	0.0532945	7.58E‐07	24.49604061
rs8066625	A	G	0.107212	0.175585	0.031912	3.84E‐08	30.27378883
rs2918299	T	C	0.166014	0.142564	0.0229551	5.45E‐10	38.57104152
rs144513708	A	G	0.018609	0.650996	0.140529	3.67E‐06	21.45975347

### 3.2 Causal effect of AD on LC

As shown in Figure 2, the IVW analysis showed a decreased risk of LUAD in AD patients (OR = 0.91, 95% CI: 0.85‐0.97, *P* = 0.007), while the estimates from the WM (OR = 0.90; 95% CI: 0.82−0.99, *P* = 0.03) and MR‐egger regression (OR = 0.86, 95% CI: 0.74−1.01, *P* = 0.073) analyses showed the same direction with the IVW method, though the *P*‐value of MR‐egger estimate was over 0.05. Additionally, using the IVW method, no causal association was found between AD and LC (OR = 0.96, 95% CI: 0.91−1.01, *P* = 0.101), LUSC (OR = 1.04, 95% CI: 0.96−1.036, *P* = 0.324), and SCLC (OR = 0.95, 95% CI: 0.82−1.10, *P* = 0.512). The results of the MR analysis are shown in Table 4.

**FIGURE 2:** Forest plot showing the results of our MR analysis. AD, atopic dermatitis; LC, lung cancer; LUAD, lung adenocarcinoma; LUSC, lung squamous cell carcinoma; SCLC, small cell lung cancer.

**TABLE 4:** Results of univariable MR analysis.

Exposure	Outcome	Method	β	SE	OR (95%CI)	*P*
AD	LC	IVW	−0.045	0.027	0.96 (0.91‐1.01)	0.101
		MR‐Egger	−0.104	0.067	0.9 (0.79‐1.03)	0.137
		Weighted median	–0.079	0.039	0.92 (0.86‐1.00)	0.040
	LUAD	IVW	−0.097	0.036	0.91 (0.85‐0.97)	0.007
		MR‐Egger	−0.150	0.080	0.86 (0.74‐1.01)	0.073
		Weighted median	−0.107	0.049	0.90 (0.82‐0.99)	0.030
	LUSC	IVW	0.042	0.043	1.04 (0.96‐1.13)	0.324
		MR‐Egger	−0.074	0.094	0.93 (0.77‐1.12)	0.441
		Weighted median	0.056	0.060	1.06 (0.94‐1.19)	0.344
	SCLC	IVW	−0.049	0.075	0.95 (0.82‐1.10)	0.512
		MR‐Egger	−0.188	0.169	0.83 (0.59‐1.15)	0.279
		Weighted median	−0.049	0.098	0.95 (0.79‐1.15)	0.616
	LUAD	IVW	‐1.226	0.619	0.29 (0.09‐0.99)	0.047
		MR‐Egger	‐3.543	1.417	0.03 (0.002‐0.465)	0.014
		Weighted median	‐1.114	0.869	0.33 (0.06‐1.80)	0.199

Abbreviations: AD, atopic dermatitis; LC, lung cancer; LUAD, lung adenocarcinoma; LUSC, lung squamous cell carcinoma; SCLC, small cell lung cancer.

### 3.3 Sensitivity analysis

Subsequently, several sensitivity analytic methods were implemented to evaluate the robustness of the preliminary results. In terms of heterogeneity, Cochran's Q test showed that there was no significant heterogeneity for total LC, LUSC, LUAD, and SCLC (all *P* > 0.05). MR‐Egger regression analysis and MR‐PRESSO test demonstrated no directional or horizontal pleiotropy in our MR analyses (all *P* > 0.05). Meanwhile, the leave‐one‐out analysis further showed the reliability of the MR results. There was no significant shift in the identified causal effect when removing a single SNP. The scatter plot, depicted in Figure 3, which highlighted the consistency of these findings. Moreover, the funnel plot and level‐one‐out analysis, depicted in Figures S1, S2 respectively, indicating the robustness of our results. The results of the sensitivity analysis are shown in Table 5.

**FIGURE 3:** Scatter plot for Mendelian randomization analysis. Note: A: AD‐LC; B: AD‐LUAD; C: AD‐LUSC; D: AD‐SCLC; AD, atopic dermatitis; LC, lung cancer; LUAD, lung adenocarcinoma; LUSC, lung squamous cell carcinoma; SCLC, small cell lung cancer.

**TABLE 5:** Sensitivity analysis of MR study.

Exposure		*P*‐value		
		Heterogeneity		Pleiotropy
	Outcome	IVW	MR‐Egger	
AD	LC	0.496	0.492	0.345
	LUAD	0.859	0.846	0.462
	LUSC	0.782	0.837	0.182
	SCLC	0.166	0.164	0.369

Abbreviations: AD, atopic dermatitis; LC, lung cancer; LUAD, lung adenocarcinoma; LUSC, lung squamous cell carcinoma; SCLC, small cell lung cancer.

## 4 DISCUSSION

To our knowledge, this is the first MR study to comprehensively assess the causal relationship between the hereditary susceptibility to AD and the risk of LC in large‐scale European population data of generalized AD. Our results drew the conclusion that genetically predicted AD in the European population might reduce the risk of developing LUAD, but not in LUSC and SCLC, which paves the way for investigating relevant molecular mechanisms, accessing clinical significance, establishing surveillance programs, and better public health decisions.

Most observational studies showed that AD was a risk factor for several cancers, like prostate cancer,^20^ non‐Hodgkin's lymphoma,^40^ kidney cancer,^16^ and non‐melanoma skin cancers,^41^ while little evidence indicated that AD was correlated with lower risk of cancers, including central nervous system cancers and pancreatic cancer.^15^ However, one recent MR study has reported that AD might increase brain cancer risk.^42^ Moreover, the identified studies on AD for LC risk were inconclusive. Castaing et al. performed a case‐control study to determine the risk of developing LC in patients with a self‐reported history of AD by questionnaire‐based interviews, and the result represented that patient‐reported history of AD reduced risk of LC (OR: 0.61; 95% CI: 0.48−0.76; *P* = 0.230).^17^ Similarly, Mariam et al. collected interview data from 1,169 LC cases and 1,486 population controls and found that subjects who reported a history of AD were inversely correlated with LC (OR: 0.73; 95% CI: 0.48−1.12).^18^ Further studies reported that LUAD was the most common histologic subtype of LC in patients with AD.^18^ Meanwhile, Juan et al. revealed that AD was positively correlated with LC risk (HR: 2.80, 95% CI: 2.59−3.03).^21^ However, the self‐reported data available on eczema were significantly inaccurate because face‐to‐face interviews might cover multiple potential confounding factors such as smoking, age, and sex. More importantly, the difficulty in distinguishing between physician‐ and self‐diagnosed AD, affects the robustness of results, and limits the ability to produce a significant inverse causality of the factors observed. Our study provides causality between the two diseases from a genetically informed perspective by using the MR method and avoiding confounders to some extent.

The results of our study are consistent with several previous studies that AD might reduce LC risk. However, AD is characterized by profound increases in inflammation responses.^43^ Emerging evidence has revealed that inflammatory conditions are associated with carcinogenesis by multiple immune evasion mechanisms.^44^, ^45^ But inflammatory conditions could also activate immune cells such as natural killer (NK) cells and cytotoxic T cells, which play crucial roles in tumor immune surveillance.^44^, ^46^ Additionally, these cells can recognize and eliminate malignant cells through direct cytotoxicity or the release of cytotoxic molecules.^44^, ^46^ Moreover, AD has specific characteristics, which establish a unique inflammatory response during disease development.^43^ AD has been hypothesized to reduce the risk of developing cancer through its overactive immune states. Pathogenesis associated with the development of AD is accompanied by the predominance of Type 2 helper T (Th2) cell immunity, highly expressed thymic stromal lymphopoietin (TSLP), and immunoglobulin E (IgE)‐mediated hypersensitivity.^47^ Th2 cells mediate effector functions by producing cytokines, resulting in the activation of immune cells.^48^ The hallmark cytokines of Th2, interleukin (IL)−4 and IL‐13 highly expressed in AD and LC patients, were associated with tumor regression by recruiting infiltrating eosinophils and macrophages, while IL‐4 and IL‐13 neutralization led to loss of the antitumor immune response.^47^, ^48^ Additionally, further mechanistic studies revealed that IL‐4 exerted an antiproliferative effect on non‐SCLC cells,^49^ while recombinant human IL‐13 significantly retard tumor growth in xenotransplantation mice.^50^ TSLP is an efficient activator of dendritic cells that promotes Th2‐mediated immune response.^51^ Systemic TSLP induction has driven a significant Th2 immunity to prevent tumorigenesis progression from atypical alveolar hyperplasia to LUAD.^52^ Moreover, serum IgE levels may be related to antitumor response in patients with atopic diseases. IgE plays an essential role in triggering immune responses to cancer cells, such as in the pancreas, colon, and rectum.^53^, ^54^, ^55^ MS4A2, the subunit of the high‐affinity IgE receptor, was associated with better prognosis in patients with LUAD, suggesting that IgE/IgE receptor signaling pathway might shape LUAD development.^56^ These experimental results strongly supported that AD might be a protective factor for LC, especially in LUAD patients.

Our study has several strengths. First, our study mimicked the RCT setting by using MR approach. When genetic variants were randomly allocated as IVs, reverse causality can be avoided. Second, we removed SNPs associated with potential confounders that might affect the results of our study, which could avoid the confounding bias of observational studies. Additionally, we only utilized GWAS data in participants with European ancestry, thereby evading the population stratification bias.

However, our study also has the following limitations. The genetic variants stem from European samples, and further studies await to generalize these findings to other races. Additionally, the present study only established a causal association between the diseases, and it awaits more studies to elucidate the specific molecular mechanisms of the inverse relationship between AD and LUAD.

## 5 CONCLUSION

This is the first MR study to comprehensively assess the causality from AD on LC. Our MR study has uncovered the underlying evidence that AD may decrease the risk of LUAD, which needs deeper mechanistic studies in the clinical setting.

## CONFLICT OF INTEREST STATEMENT

The authors declare no conflicts of interest.

## ETHICS STATEMENT

We performed the MR study by using publicly available summary statistics of GWAS studies. All studies included in cited GWAS studies have been approved by relevant ethical review board, and participants included in these studies have given informed consent. Additionally, no individual data was used in this study. Therefore, no new ethical review board approval was required.

## Supporting information

Supporting Information

Supporting Information

## Data Availability

The data that support the findings of this study are available in Integrative Epidemiology Unit‐OpenGWAS project at https://gwas.mrcieu.ac.uk/.
